The article "MicroRNA expression profile of the hippocampus in a rat model of temporal lobe epilepsy and miR-34a-targeted neuroprotection against hippocampal neurone cell apoptosis post-status epilepticus" was retracted in 2024. Reasons: duplicated images; unreliable results or conclusions; lack of ethics approval or compliance; concerns about the data.

# MicroRNA expression profile of the hippocampus in a rat model of temporal lobe epilepsy and miR-34a-targeted neuroprotection against hippocampal neurone cell apoptosis post-status epilepticus

**DOI:** 10.1186/1471-2202-13-115

**Published:** 2012-09-22

**Authors:** Kai Hu, Yuan-Yuan Xie, Chen Zhang, Dong-Sheng Ouyang, Hong-Yu Long, Dan-Ni Sun, Li-Li Long, Li Feng, Yi Li, Bo Xiao

**Affiliations:** 1 Department of Neurology, Xiangya Hospital, Central South University, Changsha, Hunan, 410008, P. R. China; 2 Department of Neurology, The Third Xiangya Hospital, Central South University, Changsha, Hunan, 410013, P. R. China; 3 Institute of Clinical Pharmacology, Central South University, Changsha, Hunan, 410078, P. R. China

**Keywords:** MiRNA, Epilepsy, Hippocampus, Apoptosis, Status epilepticus

## Abstract

**Background:**

The expression pattern and function of miRNAs in the rat model of temporal lobe epilepsy have not been well defined. Profiling miRNA expression in the rat model of temporal lobe epilepsy and investigating the function of specific miRNAs in epilepsy offers the prospect of a deeper understanding of the mechanisms of epilepsy.

**Methods:**

The lithium-pilocarpine-induced status epilepticus model and the temporal lobe epilepsy model were established in Sprague–Dawley rats. Samples were analysed to detect deregulated miRNAs in the hippocampal temporal lobe, and several of these deregulated miRNAs were confirmed by qPCR. The expression of the pro-apoptotic miR-34a was detected at 1 day, 7 days and 2 weeks post-status epilepticus and at 2 months after temporal lobe epilepsy. The antagomir of miR-34a was then utilised. The expression of miR-34a after targeting and the expression change of activated caspase-3 protein were examined. The effects of altering the expression of miR-34a and activated caspase-3 protein on neuronal survival and neuronal death or apoptosis post-status epilepticus were assessed.

**Results:**

The miRNA microarray detected 9 up-regulated miRNAs (miR-146a, -211, -203, -210, -152, -31, -23a, -34a, -27a) and 15 down-regulated miRNAs (miR-138*, -301a, -136, -153, -19a, -135b, -325-5p, -380, -190, -542-3p, -33, -144, -542-5p, -543, -296*). Some of the deregulated miRNAs (miR-146a, miR-210, miR-27a, miR-135b and miR-33) were confirmed using qPCR. Furthermore, an increase in expression of the pro-apoptotic miR-34a was demonstrated in the post-status epilepticus rat hippocampus. miR-34a was significantly up-regulated at 1 day, 7 days and 2 weeks post-status epilepticus and at 2 months after temporal lobe epilepsy. Experiments with the miR-34a antagomir revealed that targeting miR-34a led to an inhibition of activated caspase-3 protein expression, which may contribute to increased neuronal survival and reduced neuronal death or apoptosis.

The article "MicroRNA expression profile of the hippocampus in a rat model of temporal lobe epilepsy and miR-34a-targeted neuroprotection against hippocampal neurone cell apoptosis post-status epilepticus" was retracted in 2024. Reasons: duplicated images; unreliable results or conclusions; lack of ethics approval or compliance; concerns about the data.

**Conclusions:**

Our study showed the expression profile of miRNAs in the hippocampus in a rat model of temporal lobe epilepsy and an increase in the expression of the pro-apoptotic miR-34a in post-status epilepticus rats. The results show that miR-34a is up-regulated during seizure-induced neuronal death or apoptosis, and targeting miR-34a is neuroprotective and is associated with an inhibition of an increase in activated caspase-3 protein.

## Background

MicroRNAs (miRNAs) belong to a family of non-coding small RNAs and are emerging as important post-transcriptional regulators that either inhibit mRNA translation or direct target mRNA degradation [1]. They are critical for normal neuronal development and may be involved in many neurological diseases whose mechanisms remain to be explored. For example, miRNAs have important roles in gene regulatory networks involved in both brain development and adult neural plasticity [2]. miR-124a and miR-9 are able to regulate ES cell differentiation toward neuronal or glial lineages [3], and brain-specific miR-9 is critical in modulating the cellular behaviour of stem cell-derived neural progenitor cells (NPCs) [4]. Recent work by Agostini et al. found that pro-apoptotic miR-34a regulates neurite outgrowth, spinal morphology and function [5], and this work highlights the importance of miR-34a in neuronal differentiation and synaptogenesis. The studies described above are only a few examples of the involvement of miRNAs in the nervous system.

A number of studies have investigated the role of miRNAs in neurological diseases such as epilepsy. Using the pilocarpine mouse model of epilepsy, Nudelman et al. reported that neuronal activity rapidly induces transcription of the CREB-regulated miR-132 *in vivo*[6]. This was the first study to demonstrate a change in a miRNA after seizures. Sano and Henshall reported that miR-34a is up-regulated during seizure-induced neuronal death [7] and concluded that prolonged seizures cause up-regulation of miR-34a in a subfield-specific, temporally restricted manner. However, they suggested that miR-34a is most likely not important for seizure-induced neuronal death in the mouse model. Recently, Kan et al. published a study of miRNA profiles in human temporal lobe epilepsy (TLE) [8] and extended the current concepts of human mesial TLE pathogenesis to the level of miRNA-mediated gene regulation. Before Kan’s work in human TLE, Aronica et al. had also published a paper focused on a single inflammation-associated miR-146a in TLE patients [9]. More recently, the work of Henshall et al. showed that miR-134a silencing produces neuroprotective and prolonged seizure-suppressive effects [10]. One of their previous studies suggested that targeting miR-132 reduces seizure-induced neuronal death and protects the hippocampus [11]. Both studies offered a new therapeutic target for the treatment of epilepsy.

The article "MicroRNA expression profile of the hippocampus in a rat model of temporal lobe epilepsy and miR-34a-targeted neuroprotection against hippocampal neurone cell apoptosis post-status epilepticus" was retracted in 2024. Reasons: duplicated images; unreliable results or conclusions; lack of ethics approval or compliance; concerns about the data.

Epigenetic research of miRNAs associated with epilepsy is an interesting field and more findings are emerging. Most studies have focused on the function of brain-specific miRNAs following status epilepticus in the mouse model or on samples from TLE patients. The expression and functional changes of inflammation-, development- and neuronal death-associated miRNAs in epilepsy have been identified. However, studies addressing the roles of pro-apoptotic miRNAs in the mechanism of epilepsy using different models are limited. The study of miR-34a in the mouse model of epilepsy has delineated a restricted role for this pro-apoptotic miRNA. Whether miR-34a mediates seizure-induced neuronal death and how it is involved in that process in the widely used status epilepticus (SE) rat model remains to be explored.

The lithium-pilocarpine-induced SE rat model is a reliable model to study status epilepticus and temporal lobe epilepsy [12,13]. Using this model, we have detected an aberrant miRNA expression pattern in the rat hippocampus and confirmed the presence of significantly deregulated miRNAs. Because miR-34a was up-regulated in this work and in a previous study [14], we hypothesized that miR-34a is up-regulated in the rat hippocampus after status epilepticus and contributes to seizure-induced neuronal death. Our results showed that miR-34a is up-regulated in rats after status epilepticus and targeting miR-34a *in vivo* could alleviate seizure-induced neuronal death or apoptosis and increase the number of surviving neurones in the hippocampus. This research indicates the neuroprotective effects of targeting miR-34a in seizure- induced neurone cell death or apoptosis in post-status epilepticus rats.

## Methods

### Ethical statement

Animal care and sacrifice were conducted according to methods approved by the Animal Care and Use Committee, Xiangya Medical College, Central South University. All experiments were performed in accordance with the National Institute of Health Guide for the Care and Use of Laboratory Animals.

### Experimental animals, housing and husbandry

Male Sprague–Dawley (SD) rats (6–8 weeks of age, weighing 230–270 g, from the Animal Unit, Central South University, P. R. China) were used. All animals were housed in a room kept on an alternating 12 hours light–dark cycle with a controlled temperature (18°C - 25°C) and humidity (50% - 60%). Food and water were available *ad libitum*.

The article "MicroRNA expression profile of the hippocampus in a rat model of temporal lobe epilepsy and miR-34a-targeted neuroprotection against hippocampal neurone cell apoptosis post-status epilepticus" was retracted in 2024. Reasons: duplicated images; unreliable results or conclusions; lack of ethics approval or compliance; concerns about the data.

### Study design, sample size and animal allocation

The study design and animal allocation are outlined in Additional file 1. Because there was a loss of animals post-SE and some animals did not exhibit spontaneous seizures, the number of animals used in the study was somewhat larger. The study design, animal allocation and number of animals used for statistical analyses are listed in the notes of Additional file 1, and the selection of animals was random whenever it was possible. Regarding the sample size, there were 152 SD rats used in the entire study, and 102 total rats were included in the statistical analyses.

### Experimental procedures for the SE and TLE model

Lithium chloride (125 mg/kg, i.p., Sigma, USA) was injected 18–20 hours prior to the administration of pilocarpine (20 mg/kg, i.p., Sigma). The severity of convulsions was evaluated by Racine’s scale, and only those animals that were classified with a score of 4–5 were included in this study. SE was defined as the onset of continuous generalised (Racine’s scale score 4–5) seizure activity lasting no less than 40 min. Intraperitoneal pilocarpine administration (10 mg/kg) was repeated every 30 min if there were no seizures or seizure activity was classified lower than a score of 4 on Racine’s scale. The maximum dose for pilocarpine injection was 60 mg/kg. All SE rats received chloral hydrate (10%, 3 ml/kg, i.p.) to terminate epileptic attacks. The control rats received an injection of an equal amount of normal saline instead of pilocarpine. All the rats were housed in the same environment and continuous observation of animal behaviour was performed from the successful establishment of the SE model to the time of the animal’s death. The temporal lobe epilepsy rats (2 months post-SE) were identified by a frequent attack of seizures (at least two spontaneous seizures that scored 4–5 on Racine’s scale), either by direct observation or by videotape recordings. Some animals exhibiting seizures were confirmed using electroencephalogram (EEG) recordings that displayed high frequency, high amplitude, poly-spike paroxysmal discharges. The animals were killed within 5 hours of occurrence of the last spontaneous seizure. Some animals were anesthetised using chloral hydrate (10%, 5 ml/kg, ip.) and decapitated, and hippocampi were removed quickly from the brain and frozen in liquid nitrogen. Other animals were anesthetised and perfused with saline followed by 4% paraformaldehyde.

### miRNA microarray analysis

Total RNA for microarray analysis was extracted and purified using the mirVana™ miRNA Isolation Kit (Cat# AM1560, Ambion, Austin, TX, US) following the manufacturer’s instructions and checked for a RIN number to inspect RNA integrity using an Agilent Bioanalyzer 2100 (Agilent Technologies, Santa Clara, CA, US).

miRNA molecules in the total RNA were labelled by a miRNA Complete Labeling and Hyb Kit (Cat# 5190–0456, Agilent Technologies, Santa Clara, CA, US) following the manufacturer’s instructions.

The article "MicroRNA expression profile of the hippocampus in a rat model of temporal lobe epilepsy and miR-34a-targeted neuroprotection against hippocampal neurone cell apoptosis post-status epilepticus" was retracted in 2024. Reasons: duplicated images; unreliable results or conclusions; lack of ethics approval or compliance; concerns about the data.

Each slide was hybridised with 100 ng of Cy3-labeled RNA using the miRNA Complete Labeling and Hyb Kit (Cat# 5190–0456, Agilent Technologies, Santa Clara, CA, US) in hybridisation Oven (Cat# G2545A, Agilent Technologies, Santa Clara, CA, US) at 55°C and 20 rpm for 20 hours according to the manufacturer’s instructions. After hybridisation, the slides were washed in staining dishes (Cat# 121, Thermo Shandon, Waltham, MA, US) with the Gene Expression Wash Buffer Kit (Cat# 5188–5327, Agilent Technologies, Santa Clara, CA, US).

Slides were scanned using the Agilent Microarray Scanner (Cat# G2565BA, Agilent Technologies, Santa Clara, CA, US) and the Feature Extraction software 10.7 (Agilent Technologies, Santa Clara, CA, US) with the default settings. Subsequently, the microarray image information was converted into spot intensity values using the Scanner Control Software Rev. 7.0 (Agilent Technologies, Santa Clara, CA, US). The signal after background subtraction was later exported directly into the Gene Spring GX11.0 software (Agilent Technologies, Santa Clara, CA, US) for quantile normalisation. The quantile algorithm is a method of normalisation that equalises the distribution of expression values of all the samples in an experiment. The mean normalised signal from biological replicates was then used for comparative expression analysis. The unpaired *t*-test with the Benjamini-Hochberg correction was used to identify differentially expressed miRNAs between the control and epilepsy samples. The significantly deregulated miRNAs were defined as miRNAs that have p-values less than 0.05 and with an expression fold-change greater than 1.5, whether they were up-regulated or down-regulated when compared with controls. Normalised data were hierarchically clustered by gene and used to plot the heat maps.

### Quantitative real-time PCR

Total RNA was isolated using the Trizol reagent (Invitrogen, USA). Each reaction mixture of RT contained 2 μg of RNA template, 2 μL miR-RT primers, mixed with RNase-free H_2_O to 11 μL (volume A) and 5 μL RT buffer 5X, 0.5 μL 2.5 mM dNTPs, 1 μL RNase Inhibitor (40 U/μL), 0.5 μL Reverse Transcriptase (200 U/μL) (Fermentas) and RNase-free H_2_O to a total volume of 25 μL. The 11 μL volume A was mixed and centrifuged at 4°C, incubated for 10 min at 70°C and placed in an ice bath for 2 min. The 25 μL volume reactions were then incubated for 60 min at 42°C and for 10 min at 70°C.

qPCR reaction was performed using the Platinum SYBR Green qPCR Super Mix UDG (Invitrogen, USA) and ABI Mx3000P QPCR System (Stratagene). qPCR was performed in triplicates. The 20 μL qPCR reaction contained the following: 9 μL SYBR Green Mix, 2 μL miRNA RT Product, 2 μL Bulge-Loop^TM^ miRNA Forward Primer (5 μM) and 2 μL Bulge-Loop^TM^ miRNA Reverse Primer (5 μM) (RiboBio Co., Ltd, China) and RNase-free H_2_O to a final volume of 20 μL. The qPCR reactions were incubated at 95°C for 20 s, followed by 40 cycles of 95°C for 10 s, 60°C for 20 s and 70°C for 10 s and finally 95°C for 10 s, 60°C for 20 s and 95°C for 10 s.

The article "MicroRNA expression profile of the hippocampus in a rat model of temporal lobe epilepsy and miR-34a-targeted neuroprotection against hippocampal neurone cell apoptosis post-status epilepticus" was retracted in 2024. Reasons: duplicated images; unreliable results or conclusions; lack of ethics approval or compliance; concerns about the data.

The relative expression level for each miRNA was calculated by the comparative CT method. The expression of the U6 small nucleolar RNA gene was used as an internal control.

### Bioinformatics analysis

All significant differentially expressed miRNAs were analysed by bioinformatics algorithms. Potential targets of these miRNAs were predicted using the miRNA target prediction databases including TargetScan and miRanda. Functional classification was performed by Gene Ontology (GO) to determine the biological significance of these targets, and an accompanying p-value calculated by the Fisher’s Exact Test indicated which functions were over-represented in the targets. Moreover, using the KEGG pathway database, pathway analysis was performed to identify the enriched pathways of targets, and the p-value was calculated for each pathway using a hyper-geometric distribution for identification of the significance of pathways.

### miR-34a antagomir experiments

To study the potential function of miR-34a in post-SE rat hippocampal neuronal apoptosis, a miRNA antagomir strategy was adopted. We antagonised the expression of miR-34a in post-SE rat hippocampus by using an antagomir that specifically targets miR-34a. A miR-34a antagomir or an antagomir-control (miR-Ribo^TM^; RiboBio Co., Ltd., China) was dissolved in an artificial CSF (119 mmol/L NaCl, 3.1 mmol/L KCl, 1.2 mmol/L CaCl_2_, 1 mmol/L MgSO_4_, 0.5 mmol/L KH_2_PO_4_, 25 mmol/L NaHCO_3_, 5 mmol/L D-glucose, 2.2 mmol/L urea, pH 7.4) [15] at a concentration of 20 nmol/mL (1 nmol/50 μL for each rat) and infused at a very slow rate (25 μL of CSF was withdrawn for an hour and 50 μL of antagomir was infused for 2 hours) by micro- syringe into the lateral ventricle (Bregma: 0.8 mm posterior, -4.8 mm dorsoventral, -1.5 mm lateral; on the basis of the rat brain atlas of Paxinos and Watson [13]) of post-SE rats. The process began at 1 hour and ended at 4 hours after SE onset. To look for expression changes of miR-34a and its potential downstream molecules in post-SE rats that had received infusions of miR-34a antagomir and antagomir-control, rats were anesthetised using chloral hydrate (10%, 5 mL/kg, ip.) at 7 days post-SE before their hippocampal tissue was removed for detection of miR-34a expression and detection of its potential downstream molecules including activated caspase-3 protein.

The article "MicroRNA expression profile of the hippocampus in a rat model of temporal lobe epilepsy and miR-34a-targeted neuroprotection against hippocampal neurone cell apoptosis post-status epilepticus" was retracted in 2024. Reasons: duplicated images; unreliable results or conclusions; lack of ethics approval or compliance; concerns about the data.

### Western-blot analysis

The cytoplasmic extracts were separated by 12% SDS-PAGE and transferred onto a PVDF membrane using the Bio-Rad system (Bio-Rad, USA) before blocking with TBST containing 5% nonfat-milk for 2 hours at room temperature with gentle shaking. Three washing steps of 10 min each were performed after blocking and incubation with the antibodies. The primary antibody was a rabbit anti-rat activated caspase-3 polyclonal antibody (Abcam, ab2302; 1:600); β-actin expression was used as an internal control. The membrane was incubated overnight at 4°C with the primary antibody and incubated with a goat anti-rabbit IgG/HRP antibody (SCBT, sc-2030; 1:40,000) at room temperature for 1 h. The protein/antibody complexes were detected using chemiluminescence reagents (ECL) (KPL, USA). Integrated optical density (IOD) values of activated caspase-3 protein and β-actin were measured. The relative expression amount of activated caspase-3 protein was determined by the ratio of activated caspase-3 protein/β-actin.

### Immunohistochemistry

The paraffin-embedded sections were deparaffinised and rehydrated, followed by treatment with 1% hydrogen peroxide to eliminate endogenous peroxidase activity. After treatment with goat serum reagent at room temperature for 20 min, the sections were exposed to primary antibody for 2 h at room temperature and overnight at 4°C. The primary antibody was a rabbit anti-rat caspase-3 polyclonal antibody (Boster Co., China; 1:200). The sections were incubated with secondary antibody, a biotinylated goat anti-rabbit antibody (Boster Co., China; 1:200) at room temperature for 20 min, followed by incubation with a streptavidin-biotin peroxidase complex solution (Boster Co., China) at room temperature for 90 min. Subsequently, the sections were stained using diaminobenzidine, restained with hematoxylin, dehydrated and mounted. All slices were processed with a HPIAS-1000 Color Image Analysis system for imaging and analysis.

### Nissl staining and TUNEL assay

Nissl staining was performed to detect the surviving neurones. The sections were stained with 0.5% Cresyl violet (w/v) for 10 minutes before they were dehydrated and mounted with permount. The surviving neurones were only counted if they possessed intact neuronal morphology. The TUNEL assay, which detects DNA fragmentation resulting from apoptotic signalling cascades, was performed to label apoptotic neurones. It may also label cells that have suffered severe DNA damage. Therefore, the TUNEL assay is helpful in identifying seizure-induced neuronal death in our experiments. The procedures were performed according to the manufacturer’s instructions (Roche Co., Germany). TUNEL-positive cells were defined as those demonstrating blue-purple nucleic staining. The CA1 and CA3 regions of each section were captured by microscope (Olympus, Japan). Under 40 × magnification, 6 visual fields were randomly selected for each section, and the surviving neurones and the total number of cells were counted. The survival rate was calculated as follows: number of surviving neurones/total number of cells × 100%. Additionally, 6 visual fields were randomly selected to count the number of dead neuronal cells and the total number of cells. The death rate was determined as follows: number of dead neuronal cells/total number of cells × 100%. For Nissl-staining or TUNEL-assay, three sections were examined for each rat before the means were obtained for statistical analysis.

The article "MicroRNA expression profile of the hippocampus in a rat model of temporal lobe epilepsy and miR-34a-targeted neuroprotection against hippocampal neurone cell apoptosis post-status epilepticus" was retracted in 2024. Reasons: duplicated images; unreliable results or conclusions; lack of ethics approval or compliance; concerns about the data.

### Statistical methods

Statistical analysis was performed using the SPSS 13.0 software and all data were expressed as the mean ± standard deviation. Differences between multiple groups were statistically assessed by one-way ANOVA analysis, whereas differences between two groups were evaluated by the independent-samples *t*-test. For statistical analysis, *p* < 0.05 was considered to be statistically significant.

## Results

### Animal number analysed

The number of animals in each group included in each analysis is reported in Additional file 1. Absolute numbers were used in the report. The animals and data not included in the analysis, as well as their reasons, are also clearly mentioned in the notes of Additional file 1.

### miRNA expression profile of the hippocampus in a rat model of TLE

The Agilent Rat miRNA microarray used in this study covered over 350 rat miRNAs detected so far, and the sequence information is based on the Sanger miR-Base version 12.0. The miRNA microarray scanned images and the normalised primary microarray data are shown in Additional files 2 and 3, respectively. The cluster and heatmap of all detected rat miRNAs in this study are plotted and shown in Figure 1. The miRNA microarray differential analysis resulted in 24 significantly deregulated miRNAs as shown in Table 1, and the heatmap of these 24 aberrantly expressed miRNAs is plotted and shown in Figure 2. Among the 24 significantly deregulated miRNAs, 9 miRNAs (miR-146a, -211, -203, -210, -152, -31, -23a, -34a, -27a) were up-regulated and 15 miRNAs (miR-138*, -301a, -136, -153, -19a, -135b, -325-5p, -380, -190, -33, -542-3p, -144, -542-5p, -543, -296*) were down-regulated (differentially expressed miRNAs were defined by a fold-change >1.5, either up-regulated or down-regulated; *p <0.05).

The article "MicroRNA expression profile of the hippocampus in a rat model of temporal lobe epilepsy and miR-34a-targeted neuroprotection against hippocampal neurone cell apoptosis post-status epilepticus" was retracted in 2024. Reasons: duplicated images; unreliable results or conclusions; lack of ethics approval or compliance; concerns about the data.

**Figure 1:** **The heatmap of all rat hippocampal TLE miRNAs.** Rows represent individual genes, and columns represent individual samples. The high (red), average (black) and low (green) expression levels are depicted by the colourgram (n = 6 for TLE rats and n = 6 for control).

**Table 1:** The 24 significantly deregulated miRNAs in the TLE rat hippocampus

**MicroRNA**	**Fold change**	**Regulation**	***p*value**
rno-miR-146a	2.6958885	up	1.258E-02
rno-miR-211	2.610144	up	1.376E-02
rno-miR-203	2.109093	up	2.367E-02
rno-miR-210	1.8106444	up	1.999E-02
rno-miR-152	1.7704262	up	8.17E-04
rno-miR-31	1.6925983	up	3.811E-03
rno-miR-23a	1.5156718	up	7.727E-03
rno-miR-34a	1.4842122	up	2.398E-02
rno-miR-27a	1.4451101	up	1.133E-02
rno-miR-138*	1.5289445	down	3.512E-02
rno-miR-301a	1.5327321	down	7.925E-03
rno-miR-136	1.5330569	down	4.166E-03
rno-miR-153	1.5534221	down	1.826E-02
rno-miR-19a	1.6450298	down	1.832E-02
rno-miR-135b	1.657749	down	2.853E-02
rno-miR-325-5p	1.8619193	down	4.587E-02
rno-miR-380	1.8745395	down	1.176E-02
rno-miR-190	1.8834999	down	1.528E-02
rno-miR-542-3p	1.8835889	down	7.955E-03
rno-miR-33	1.9224428	down	3.279E-03
rno-miR-144	1.9507241	down	4.969E-02
rno-miR-542-5p	2.2845843	down	5.943E-03
rno-miR-543	3.0247948	down	1.067E-03
rno-miR-296*	3.0831256	down	2.85E-06

***Notes:*** The Agilent rat miRNA microarray identified 24 significantly deregulated miRNAs (fold change >1.5, expression either upregulated or down-regulated; *p <0.05) in the hippocampus of the TLE rat when compared with the control (n = 6 for each group).

**Figure 2:** **The heatmap of differentially expressed hippocampal miRNAs in the TLE rat.** The 24 significantly deregulated miRNAs have been rearranged in this heatmap, where 9 up-regulated and 15 down-regulated miRNAs are clearly displayed (n = 6 for TLE rats and n = 6 for control).

### miRNA confirmation using qPCR

To validate the altered expression of miRNAs as detected by miRNA microarray, miR-146a, miR-210, miR-27a, miR-135b and miR-33 were selected for confirmation by quantitative real-time PCR. The results were consistent with that of the microarray analysis. As seen in Figure 3, the expression levels of miR-146a, miR-210 and miR-27a were up-regulated, while the expression levels of miR-135b and miR-33 were down-regulated (*p < 0.05).

**Figure 3:** **The quantitative real-time PCR validation for some expression-altered miRNAs.** The five differentially expressed miRNAs (miR-146a, miR-210, miR-27a, miR-135b and miR-33) in the TLE rat hippocampus as detected by the Rat miRNA microarray were confirmed using qPCR (Data are presented as the mean ± SEM, *p <0.05; n = 6/TLE rats, n = 6/control). White bars: control; Black bars: experimental.

The article "MicroRNA expression profile of the hippocampus in a rat model of temporal lobe epilepsy and miR-34a-targeted neuroprotection against hippocampal neurone cell apoptosis post-status epilepticus" was retracted in 2024. Reasons: duplicated images; unreliable results or conclusions; lack of ethics approval or compliance; concerns about the data.

### Bioinformatics analysis

There were 1315 and 8810 target genes predicted by microRNA target prediction databases TargetScan and miRanda. The GO terms significantly over-represented in deregulated miRNA targets are listed in Figure 4, where the percent and enrichment test *p* values for each GO term are indicated. Some of the top KEGG pathways important in the molecular mechanism of epilepsy are significantly over-represented among the deregulated miRNA targets and are listed in Additional file 4. The signalling pathways enriched in temporal lobe epilepsy are consistent with previous studies of the molecular portrait of basic epilepsy mechanisms using whole transcriptome analysis of the hippocampus [16].

**Figure 4:** **GO terms significantly over-represented among the deregulated miRNA targets are shown.** The percent and enrichment test *p* value for each GO term are indicated in this figure.

### miR-34a expression post-SE

Expression of the pro-apoptotic miR-34a in the rat hippocampus was examined. The time points chosen for miR-34a detection were 1 day, 7 days, 2 weeks post-SE and 2 months (TLE). The expression pattern of miR-34a is shown in Figure 5. Pro- apoptotic miR-34a was significantly increased in post-SE rat hippocampus at all four time points chosen (*p <0.05). Its over-expression was notably higher at 1 day, 7 days and 2 weeks post-SE before it went down to a lower level at 2 months in temporal lobe epilepsy, although it was still markedly higher than control.

**Figure 5:** **The expression pattern of miR-34a is shown.** The study time points were 1 day, 1 week, 2 weeks (post-SE) and 2 months (TLE). The pro-apoptotic miR-34a displayed increased expression at all four time points chosen (Data are presented as the mean ± SEM, *p <0.05; n = 6 for each group), when compared with control.

### miR-34a antagomir outcomes

miR-34a antagomir treatment significantly reduced the expression of miR-34a in the rat hippocampus at 7 days post-SE (*p <0.05), when compared with the miR-34a antagomir-control-treated group (Figure 6A). Furthermore, the miR-34a antagomir specifically targeting miR-34a did not exert any antagonising effects on other miRNAs in the rat hippocampus at 7 days post-SE (data not shown). The use of miRNA antagomirs is a successful strategy for studies of miRNA function, both *in vivo* and *in vitro*, because antagomirs effectively and specifically inhibit endogenous miRNAs by causing their degradation with effects that persist at least one week or longer (Instructions for miR-Ribo^TM^ Antagomir and Antagomir-control; RiboBio Co., Ltd., China).

The article "MicroRNA expression profile of the hippocampus in a rat model of temporal lobe epilepsy and miR-34a-targeted neuroprotection against hippocampal neurone cell apoptosis post-status epilepticus" was retracted in 2024. Reasons: duplicated images; unreliable results or conclusions; lack of ethics approval or compliance; concerns about the data.

**Figure 6:** **The results of the miR-34a antagomir experiment.** Inhibition of miR-34a expression by the miR-34a antagomir at 7 days post-SE in the rat hippocampus is shown in. **A**. The miR-34a antagomir significantly inhibited the expression of miR-34a in the post-SE rat hippocampus when compared with the antagomir-control (Data are presented as the mean ± SEM, *p < 0.05; n = 6 for each group). The expression of activated caspase-3 protein in the post-SE rat hippocampus both before and after miR-34a antagomir/antagomir-control treatments as detected by western blot analysis is shown in **B**. Western blot detected an up-regulation in the expression of activated caspase-3 protein at 7 days post-SE in the rat hippocampus, when compared with control (*p <0.05, n = 6 for each group). The expression of activated caspase-3 protein at 7 days post-SE in the rat hippocampus, however, decreased in the miR-34a antagomir-treated group, when compared with the antagomir-control-treated group (**p < 0.05, n = 6 for each group).

### Alteration of activated caspase-3 expression

The Western blot results demonstrated an up-regulation of activated caspase-3 protein expression at 7 days post-SE in the rat hippocampus, when compared with the control (*p <0.05) (Figure 6B). Moreover, the expression level of activated caspase-3 protein at 7 days post-SE in the rat hippocampus decreased after miR-34a antagomir treatment, when compared with the miR-34a antagomir-control-treated group (*p <0.05) (Figure 6B). Immunohistochemistry confirmed the western blot results shown in Figure 7, where the activated caspase-3 protein was significantly over-expressed in the post-SE rat hippocampal CA1 region and CA3 regions (Figure 7F and Figure 7J) when compared with the control (Figure 7E and Figure 7I). Moreover, activated caspase-3 protein expression was significantly down-regulated in the post-SE rat hippocampal CA1 and CA3 regions after miR-34a antagomir treatment (Figure 7G and Figure 7K) when compared with the antagomir-control-treated group (Figure.7H and Figure 7L).

**Figure 7:** **Activated caspase-3 protein in the post-SE rat hippocampus.** Overview: **A-D**; CA1 region: **E-H**; CA3 region: **I-L**. Scale bars: 300 μm (**A-D**); 30 μm (**E-L**).

### Alterations in neuronal survival and neuronal death

Nissl-staining was performed to detect surviving neurones, and the TUNEL-assay was used to label apoptotic neurones by detecting the DNA fragmentation that results from apoptotic signalling cascades. It may also label cells that have suffered severe DNA damage. TUNEL is therefore helpful for identifying seizure-induced neuronal death in our experiments.

The article "MicroRNA expression profile of the hippocampus in a rat model of temporal lobe epilepsy and miR-34a-targeted neuroprotection against hippocampal neurone cell apoptosis post-status epilepticus" was retracted in 2024. Reasons: duplicated images; unreliable results or conclusions; lack of ethics approval or compliance; concerns about the data.

In the post-SE rat hippocampus, neuronal survival decreased, whereas neuronal death increased (at 7 days post-SE) (Table 2, Figure 8 and Figure 9). As seen, neuronal survival was reduced in the post-SE rat hippocampal CA1 and CA3 regions (Figure 9F and Figure 9J; Figure 9E and Figure 9I as control), and neuronal death increased in the CA1 and CA3 regions (Figure 8F and Figure 8J; Figure 8E and Figure 8I as controls).

**Table 2:** Neuronal death (apoptosis) and neuronal survival at 7 days post-SE in the rat hippocampus

**Neurones**	**Control**		**Epilepsy**		**Antagomir**		**Antagomir-control**	
	**CA1**	**CA3**	**CA1**	**CA3**	**CA1**	**CA3**	**CA1**	**CA3**
Percent Death	17.91 ± 4.78%	20.57 ± 5.02%	48.86 ± 12.39% ^a^	40.39 ± 11.42% ^a^	30.49 ± 8.91% ^b^	24.80 ± 5.80% ^b^	49.35 ± 12.74%	40.69 ± 10.97%
Percent Survival	88.15 ± 10.02%	78.89 ± 8.92%	47.32 ± 11.93% ^a^	51.25 ± 14.80% ^a^	72.81 ± 10.60% ^b^	68.28 ± 11.54% ^b^	46.26 ± 9.50%	52.05 ± 14.70%

***Notes:*** In rat hippocampal CA1 and CA3 regions, the number of dead neurones or apoptotic cells was significantly increased and the number of surviving neurones was markedly decreased at 7 days post-SE, as detected by the TUNEL-assay and Nissl-staining (^*a*^*P < 0.01, epilepsy vs control, n = 6 /group*). In the same regions, however, neuronal death or apoptosis was decreased and neuronal survival was increased significantly after miR-34a antagomir or antagomir-control treatment (^*b*^*P < 0.01, miR-34a antagomir vs antagomir-control, n = 6 /group*). The survival rate is determined by the number of surviving neurones/ number of total cells × 100%, whereas the neuronal death or apoptotic rate is determined by the number of dead neurones or apoptotic cells/ number of total cells × 100%.

**Figure 8:** **Neurone cell death or apoptosis visualised by the TUNEL-assay in the post-SE rat hippocampus.** Overview: **A-D**; CA1 region: **E-H**; CA3 region: **I-L**. Scale bars: 300 μm (**A-D**); 30 μm (**E-L**).

**Figure 9:** **Neurone survival visualised by Nissl-staining in the post-SE rat hippocampus.** Overview: **A-D**; CA1 region: **E-H**; CA3 region: **I-L**. Scale bars: 300 μm (**A-D**); 30 μm (**E-L**).

miR-34a antagomir treatment had an inhibitory effect on activated caspase-3 protein expression and led to an increase in neuronal survival as well as a decrease in seizure-induced neuronal death at 7 days post-SE in the rat hippocampus (Table 2, Figure 8 and Figure 9). The number of surviving neurones was markedly increased in the CA1 and CA3 regions (Figure 9G and Figure 9K; Figure 9H and Figure 9L as controls) when compared with the antagomir-control-treated group. Additionally, there was a significant decrease in neuronal cell death after miR-34a antagomir treatment in the post-SE rat hippocampal CA1 and CA3 regions (Figure 8G and Figure 8K; Figure 8H and Figure 8L as controls) when compared with the control.

The article "MicroRNA expression profile of the hippocampus in a rat model of temporal lobe epilepsy and miR-34a-targeted neuroprotection against hippocampal neurone cell apoptosis post-status epilepticus" was retracted in 2024. Reasons: duplicated images; unreliable results or conclusions; lack of ethics approval or compliance; concerns about the data.

## Discussion

Because a number of previous studies have investigated the role of miRNAs in epilepsy [6-11,14,17], it is important to provide a discussion of our own data in light of previously published profiles and results. Different models may yield different study outcomes, and comparisons of results between different or even the same models are necessary. Similar to our study, Song et al. used the classical status epilepticus rat model and reported differential expression of miRNAs in the hippocampus in a rat model of TLE [17]. Yet, the number of samples used for miRNA microarray analysis (TLE rats = 3, control rat = 1) in their study did not strictly conform to the limits needed for statistical analysis. Furthermore, the standards to screen differentially expressed miRNAs in their study (fold-change: three ratios >1 plus at least two ratios >1.5 for up-regulated miRNAs; three ratios *<*1 plus at least two *<*0.67 for down-regulated miRNAs) did not meet the stringent conditions of the method for analysing miRNA microarray raw data; the overall inclusion of all data, where miRNA signal intensities and all microarray values are integrated for statistics, appears to be preferable. Therefore, we investigated the miRNA expression profile of TLE in the rat hippocampus using a more rigorous design of animal numbers (TLE rats = 6, control = 6) and method of analysing microarray raw data. The results from our study were different to some extent from Song’s report. There were some common differentially expressed miRNAs in the two studies; e.g., both detected an up-regulation of the inflammation-associated miR-146a and the apoptotic miR-23a. However, many differentially expressed miRNAs detected varied between the two studies. For example, the pro-apoptotic miR-34a was detected in our study as a significantly deregulated miRNA, and further investigation of the expression and function of miR-34a in the mechanism of epilepsy was performed.

To extend the animal studies to human research, Kan et al. recently detected miRNA profiles in human TLE and reported marked aberrant expression of miRNAs in mTLE patients [8]. In their study, autopsy control patients and two mTLE patient groups were compared, and segregated miRNA signatures for three different patient groups were revealed. Analysis of the changes of individual miRNAs identified 165 miRNAs with up- or down-regulated expression, and 51 of these miRNAs exhibited a fold change >2.0. Interestingly, the significantly deregulated inflammation-associated miR-146a detected in a TLE patient by Aronica et al. [9] and in the rat model of TLE by Song et al. [17] and our research was not identified in Kan’ work. This could be due to different standards for the selection of TLE patients or varied criteria for the surgery selection of TLE patients. In addition, different standards to screen for significantly deregulated miRNAs may also contribute to a difference in results. Because the human species exhibits a much larger pool of miRNAs than rats, it is natural that miRNA profiling in human TLE patients may result in a larger number of differentially expressed miRNAs than in rats with TLE. Some deregulated miRNAs were identified both in the TLE patients of Kan’s work and in our rat TLE model, such as miR-27a, miR-190, miR-203 and miR-301a. Moreover, Kan’s findings suggest that miRNA changes in mTLE affect the expression of immunomodulatory proteins and further facilitate immune responses. Accordingly, the KEGG pathway analysis of differentially expressed miRNAs in our research also identified that pathways in signal transduction and immune system were significantly enriched. They are consistent with opinion that immune cells and their inflammatory mediators play an important role in the pathophysiology of seizures and epilepsy [18].

The article "MicroRNA expression profile of the hippocampus in a rat model of temporal lobe epilepsy and miR-34a-targeted neuroprotection against hippocampal neurone cell apoptosis post-status epilepticus" was retracted in 2024. Reasons: duplicated images; unreliable results or conclusions; lack of ethics approval or compliance; concerns about the data.

Studies by the Henshall group [10,11] identified the functions of several miRNAs in epilepsy by using mouse models. In a recent paper, Henshall et al. reported that miR-134, a miRNA implicated in the control of dendritic spine morphology, was up-regulated in a mouse model of status epilepticus, and silencing of miR-134 expression reduced neurone dendrite spine density and rendered mice refractory to seizures [10]. The Henshall group also reported that the expression level of another miRNA, miR-132, was increased following status epilepticus. Targeting miR-132 *in vivo* depleted miR-132 levels in the mouse hippocampus and reduced the seizure-induced neuronal death [11]. Furthermore, Sano et al. reported miR-34a up-regulation during seizure-induced neuronal death in a mouse model [7] and concluded that miR-34a up-regulation in subfield-specific, temporally restricted manner is most likely not important for seizure-induced neuronal death. The strategy of these studies commonly includes the selection of a target miRNA followed by expression analysis and the use of an antagomir. The target miRNAs chosen were mainly brain-specific and possess functions in either dendritic spine morphogenesis or neuronal cell death, as these aspects are important factors for the development of epilepsy. The immune response and astrocytes have also been identified to play a role in epileptogenesis, yet miRNA functional studies concerning this aspect of the mechanism of epilepsy are few and more studies are needed.

The article "MicroRNA expression profile of the hippocampus in a rat model of temporal lobe epilepsy and miR-34a-targeted neuroprotection against hippocampal neurone cell apoptosis post-status epilepticus" was retracted in 2024. Reasons: duplicated images; unreliable results or conclusions; lack of ethics approval or compliance; concerns about the data.

The Sano study did not detect a protective effect of the miR-34a antagomir in the kainic acid-induced status epilepticus mouse model, although they showed an up-regulation of miR-34a in hippocampal subfields after status epilepticus. This is somewhat different from our results, as we have not only found an up-regulation of miR-34a in the post-status epilepticus rat hippocampus but also detected a neuro-protective effect of targeting miR-34a during seizure-induced neuronal death. The reasons for the difference in these results are multi-faceted, but the most important reason is likely due to the different epilepsy models used. There are various animal models with chronic brain dysfunction that are thought to reflect processes underlying human epilepsy. These chronic models of epilepsy include the kindling model of TLE and post-status epilepticus models of TLE. Pilocarpine and kainate models replicate features of human TLE and can be used as animal preparations for understanding the basic mechanisms of epileptogenesis [13]. However, differences between the models, species and strains do exist in that the processes underlying epileptogenesis and the extent of neuronal damage differs [19]. Furthermore, the degree to which miR-34a can induce apoptosis may vary between different models. For example, there is evidence for miR-34a having varying effects in the promotion of apoptosis [20,21]. As up-regulation of miR-34a caused by prolonged seizures *in vivo* has already been shown, we propose that miR-34a may have a more important role in the lithium- pilocarpine-induced status epilepticus in rats. In this model, neuronal injury leads to miR-34a up-regulation, and the protective effect of the miR-34a antagomir in our study may be related to the ability of miR-34a to induce apoptosis in post-status epilepticus rats. Because seizure-induced neuronal death may be more prominent when miR-34a has much stronger pro-apoptotic function, targeting miR-34a may result in subsequent neuroprotective effects.

The potential mechanism of miR-34a regulation of downstream targets needs further mention. miR-34a up-regulation in a transgenic mice model of Alzheimer’s disease resulted in a higher expression level of activated caspase-3 protein by inhibiting bcl-2 translation, suggesting that bcl-2 is an important target for miR-34a [22]. This is consistent with results from previous studies that identified bcl-2 as a miR-34a target [23-26]. Because abnormal expression of miR-34a may contribute to the pathogenesis of Alzheimer’s disease, it is speculated that seizure-induced up-regulation of miR-34a may also play a role in the pathophysiology of epilepsy, at least in part by affecting bcl-2 expression. Prolonged experimental seizures can cause apoptosis and activate caspases and bcl-2 family proteins [27]. These apoptosis-associated genes may contribute to mechanisms underlying the development and maintenance of epilepsy, and modulating these genes can alter hippocampal damage after seizures. miR-34a as an epigenetic factor may play a role in modulating apoptosis-related genes such as bcl-2 and the caspases after status epilepticus. We focused on the effects of antagonising miR-34a on the expression of the end-phase apoptosis executor, the caspase-3 gene, to show that pro-apoptotic miR-34a and caspase-3 expression levels are related. Seizure-induced neuronal death was less prominent after treatment with the miR-34a antagomir in the post-status epilepticus rat hippocampus. What accounts for the neuroprotective effect is most likely due to a milder inhibitory effect of reduced miR-34a expression on bcl-2 translation, resulting in a lowered expression level of activated caspase-3 protein and subsequent reduction in seizure-induced neuronal death.

The article "MicroRNA expression profile of the hippocampus in a rat model of temporal lobe epilepsy and miR-34a-targeted neuroprotection against hippocampal neurone cell apoptosis post-status epilepticus" was retracted in 2024. Reasons: duplicated images; unreliable results or conclusions; lack of ethics approval or compliance; concerns about the data.

## Conclusions

In conclusion, our results demonstrate the expression profile of miRNAs in the hippocampus in a rat model of TLE and the pattern of expression increase of the pro-apoptotic miR-34a in post-SE rats. This study also demonstrated up-regulation of miR-34a in seizure-induced neuronal death or apoptosis and showed the neuro-protective effect of targeting miR-34a. The latter may be related to a lowered expression level of the activated caspase-3 protein. The present research provides insight into the involvement of miRNAs in the mechanism of epilepsy.

## Abbreviations

MiRNAs: MicroRNAs; NPCs: Neural progenitor cells; AEDs: Anti-epileptic drugs; SE: Status epilepticus; TLE: Temporal lobe epilepsy; EEG: Electroencephalogram; GO: Gene ontology; XIAP: X-linked inhibitor of apoptosis protein.

## Competing interests

The authors declare that they have no competing interests.

## Authors’ contributions

KH contributed to the study design and established the SE model, extracted the miRNAs and contributed in paper writing. YYX contributed to western blot analysis, immnohistochemistry, TUNEL-assay and Nissl-staining. CZ and HYL carried out the quantitative real-time PCR. DSO contributed to the statistical analyses and paper writing. DNS and LLL performed the bioinformatic analysis. LF and YL carried out the miRNA antagomir experiment. BX contributed in study design, supervised the study and contributed in paper writing. All authors read and approved the final manuscript.

The article "MicroRNA expression profile of the hippocampus in a rat model of temporal lobe epilepsy and miR-34a-targeted neuroprotection against hippocampal neurone cell apoptosis post-status epilepticus" was retracted in 2024. Reasons: duplicated images; unreliable results or conclusions; lack of ethics approval or compliance; concerns about the data.

## Supplementary Material

Additional file 1 **Study design, sample size and animal allocation.** The experiments, grouping design, sample size and animal number for statistical analyses are detailed in this file. Click here for file

Additional file 2 **Agilent Rat miRNA microarray scanned images.** The 12 Agilent Rat miRNA microarray scanned images are shown in this file. Click here for file

Additional file 3 **Agilent Rat miRNA microarray raw data.** The 12 Agilent Rat miRNA microarray raw data are shown in this file. Click here for file

Additional file 4 **The KEGG pathway analysis results.** The significantly enriched pathways of deregulated miRNA targets, as predicted by the KEGG pathway database, are shown in this file. Click here for file
